The article "A Weighted Error Distance Metrics (WEDM) for Performance Evaluation on Multiple Change-Point (MCP) Detection in Synthetic Time Series" was published in 2022. Journal: Comput Intell Neurosci.

# A Weighted Error Distance Metrics (WEDM) for Performance Evaluation on Multiple Change-Point (MCP) Detection in Synthetic Time Series

**DOI:** 10.1155/2022/6187110

**Published:** 2022-03-24

**Authors:** Jin Peng. Qi, Fang. Pu, Ying. Zhu, Ping. Zhang

**Affiliations:** ^1^College of Information Science & Technology, Donghua University, Shanghai 201620, China; ^2^Informationization Office, Donghua University, Shanghai 201620, China; ^3^HNSW Health Pathology East Genetics Level 4, Campus Centre, Prince of Wales Hospital Randwick, Randwick, NSW, Australia; ^4^Menzies Health Institute Queensland, Griffith University, Southport, Queensland, Australia

## Abstract

Change-point detection (CPD) is to find abrupt changes in time-series data. Various computational algorithms have been developed for CPD applications. To compare the different CPD models, many performance metrics have been introduced to evaluate the algorithms. Each of the previous evaluation methods measures the different aspects of the methods. Based on the existing weighted error distance (WED) method on single change-point (CP) detection, a novel WED metrics (WEDM) was proposed to evaluate the overall performance of a CPD model across not only repetitive tests on single CP detection, but also successive tests on multiple change-point (MCP) detection on synthetic time series under the random slide window (RSW) and fixed slide window (FSW) frameworks. In the proposed WEDM method, a concept of normalized error distance was introduced that allows comparisons of the distance between the estimated change-point (eCP) position and the target change point (tCP) in the synthetic time series. In the successive MCPs detection, the proposed WEDM method first divides the original time-series sample into a series of data segments in terms of the assigned tCPs set and then calculates a normalized error distance (NED) value for each segment. Next, our WEDM presents the frequency and WED distribution of the resultant eCPs from all data segments in the normalized positive-error distance (NPED) and the normalized negative-error distance (NNED) intervals in the same coordinates. Last, the mean WED (MWED) and MWTD (1-MWED) were obtained and then dealt with as important performance evaluation indexes. Based on the synthetic datasets in the Matlab platform, repetitive tests on single CP detection were executed by using different CPD models, including ternary search tree (TST), binary search tree (BST), Kolmogorov–Smirnov (KS) tests, *t*-tests (T), and singular spectrum analysis (SSA) algorithms. Meanwhile, successive tests on MCPs detection were implemented under the fixed slide window (FSW) and random slide window (RSW) frameworks. These CPD models mentioned above were evaluated in terms of our WED metrics, together with supplementary indexes for evaluating the convergence of different CPD models, including rates of hit, miss, error, and computing time, respectively. The experimental results showed the value of this WEDM method.

The article "A Weighted Error Distance Metrics (WEDM) for Performance Evaluation on Multiple Change-Point (MCP) Detection in Synthetic Time Series" was published in 2022. Journal: Comput Intell Neurosci.

## 1. Introduction

Change-point (CP) detection is the application of core techniques to detect abrupt changes in properties of time-series data. It has been widely studied in many real-world problems, such as atmospheric and financial analyses [1], fault detection in engineering systems [2, 3], changes detection in a variance of oceanographic time series [4], genetic time-series analyses [5], and online detection of steady-state operation [6]. For example, the usage of this method to detect abnormal patterns in ECG and EEG signals may also be beneficial [4, 7–15]. This application would allow appropriate staff to be alerted of abrupt changes in a patient's medical situation and to provide on-time treatment [16, 17]. In addition, CPD models can be tightly combined with some nonlinear modeling approaches and their applications, such as classification of human hand movements [18], degradation signal for prognostic improvement [19], real-life hand prosthetic control [20], single-channel surface electromyography (sEMG)-based control [21]. CPD models utilize algorithms that cover the fields of data mining, statistics, and computer science, including parametric and nonparametric methods [8, 22–27]. Each CPD algorithm can be assessed from the aspect of detection accuracy, computational cost, or whether it can be a real-time detection.

Many performance metrics have been introduced to evaluate CPD algorithms based on the type of decisions they make [28]. Aminikhanghahi and Cook [29] reviewed the performance evaluation methods commonly used for CPD models. The evaluation can be based on a yes/no decision whether the resultant change point was detected within a certain distance from the actual change point. In this case, the CPD model can be treated as a binary classification model and can be evaluated with the usual measures, such as accuracy, sensitivity, specificity, or ROC curve [30, 31]. For real applications, for example, clinical decision-making, cut-offs applied to the model outcomes can be adjusted to achieve different sensitivity and specificity [32]. However, when the difference in time between the resultant eCP and the actual tCP represents the measure of CPD performance, then the evaluation of these algorithms is not as straightforward as for the binary classification. There is no single label against which the performance of the algorithm can be measured. A few useful metrics consider the distance between the eCP and the tCP to measure CPD method performance. These metrics include mean absolute error (MAE), mean squared error (MSE), mean signed difference (MSD), root mean squared error (RMSE), and normalized root mean squared error (NRMSE). Of these, except NRMSE normalizes the unit size of the predicted value and facilitates a more direct comparison of error between different datasets, the other methods measure only the absolute distances between the eCP and the tCP. However, even NRMSE does not count the difference between the situations when the eCP is before and after the actual tCP. It also fails to consider the relative position of the tCP within the total length of the time-series sample.

The article "A Weighted Error Distance Metrics (WEDM) for Performance Evaluation on Multiple Change-Point (MCP) Detection in Synthetic Time Series" was published in 2022. Journal: Comput Intell Neurosci.

In our previous studies [33], a preliminary WED method was proposed for evaluating a CPD model for single change-point detection. In this existing method, a concept of weighted error distance (WED) is introduced for counting a normalized error distance between each pair of the resultant eCPs and the actual tCPs, and then the performance of different CPD models is ranked by the averaged WED accordingly [33]. In this study, a novel WEDM method is proposed to compare the overall performance of CPD models for MCPs detection on multiple data segments in a time series with different data features. Based on the previous WED measure, a concept of normalized error distance was introduced in this WEDM method, that allows comparisons of the distance between the estimated change-point (eCP) position and the target change point (tCP). During the successive MCPs detection, the proposed WEDM method first divides the original sample into a series of data segments in terms of assigned tCPs, and then counts a normalized error distance (NED) value for each segment. Then, our WEDM presents the frequency and WED distribution of the resultant eCPs from all data segments in the normalized positive-error distance (NPED) and the normalized negative-error distance (NNED) intervals in the same coordinates. Last, the mean WED (MWED) and MWTD (1-MWED) were calculated and dealt with as important performance indexes. Based on the synthetic datasets in the Matlab platform, both repetitive tests on single CP detection and successive test on MCPs detection were executed by using different CPD models, including ternary search tree (TST) [8, 34], binary search tree (BST) [15, 24], Kolmogorov–Smirnov (KS) tests [22, 25], *t*-tests (T) [23, 35], and singular spectrum analysis (SSA) algorithms [36] recorded in our previous studies [22, 37]. Meanwhile, these CPD models above were evaluated under the random slide window (RSW) [8, 38, 39] and fixed slide window (FSW) frameworks [40–44] in terms of our WEDM and supplementary indexes including the rates of hit, miss, error, and computing time, respectively. The experimental results showed the value of this WEDM method.

The article "A Weighted Error Distance Metrics (WEDM) for Performance Evaluation on Multiple Change-Point (MCP) Detection in Synthetic Time Series" was published in 2022. Journal: Comput Intell Neurosci.

## 2. Methods

In this part, the proposed WEDM is theoretically illuminated in the following steps. First, the diagnosed sample is divided into a series of data segments according to the assigned target MCPs. Second, a normalized error distance (NED) is calculated by comparing the distance between the resultant eCP position and the actual tCP within each data segment. Third, the frequency and WED distribution of the resultant eCPs detected from all segments are presented across the normalized positive-error distance (NPED) and the normalized negative-error distance (NNED) intervals in the same coordinates. Last, the metrics of mean WED (MWED) and mean WTD (MWTD) are given to efficiently evaluate a CPD model for MCPs detection on a series of data fluctuations in an identical time series.

### 2.1. Data Segmentation

Suppose a time-series signal *X*={*X*_1_,…, *X*_*i*_,…, *X*_*N*_} can be observed as a trajectory of a multiple data distribution process, in which the segment *X*_*i*_ is defined by the following equation:

(1) $$\begin{array}{c} X_{i}=f_{i}\left(t\right)+\varepsilon_{i}, \end{array}$$

where *t*∈{ *t*_*i*−1_+1,..., *t*_*i*_}, 0< *i* ≤ *M*, and *f*_*i*_  ∈ {*f*_1_,…, *f*_*M*_} is a deterministic and piece-wise function of one-dimensional signal with change points (satisfying  *f*_*i*_  ≠ *f*_*i*+1_, and *i* = 1,…, *M*−1 for insuring that abrupt changes occur), and *M*∈{1, 2,…, *n*} is the number of data segment regimes and therefore *M*−1 is the number of abrupt changes, 0 = *t*_0_ < *t*_1_< ···< *t*_*i*_ <···< *t*_*M*_ = *n*. The number *M*−1 and locations *η*_1_,. . ., *η*_*M*−1_ of change points in the process are supposed to be unknown. The sequence (*ε*_*i*_)_*i*_ _∈_ _*N*_ is assumed to be random white noise and such that E(*ε*_*i*_) is exactly or approximately zero. In the simplest case, (*ε*_*i*_)_*i*_ _∈_ _*N*_ is modeled as *i*.*i*.*d*., but can also follow more complex time-series distributions.

Consider an observed time-series signal *X*={*X*_1_,…, *X*_*i*_,…, *X*_*N*_} with *M*−1 change points mentioned above, one-part time series *X*′={*X*_*s*_,…, *X*_*j*_,…, *X*_*e*_} with a size of *N*′ is selected from *X*, 1 ≤ *s* < *j* < *e* ≤ *N*, and  1 < *N*′ ≤ *N*. Suppose a set of target MCPs *tMCP* set={*tCP*_1_,…, *tCP*_*n*_} is contained within *X*′, and 1 ≤ *n* ≤ *M* − 1. In the proposed WEDM method, the diagnosed data sample *X*′ is first divided into a series of data segments according to different target CP positions in the *tMCP* set. The process of data segmentation is described below (Figure 1):

(1) For each *tCP*_*i*_ to be diagnosed in the *tMCP* set, the data segment *Seg*_*i*_ can be denoted as follows:
  (2) $$\begin{array}{c} Seg_{i}=\left\{mtCP_{i-1},\ldots ,\;tCP_{i}\ldots ,mtCP_{i}\;\right\}, \end{array}$$
   where 1 < *i* < *n* and 1 < *n* < *N*′, and two endpoints *mCP*_*i*−1_ and *mCP*_*i*_ in *Seg*_*i*_ are formulated as follows:
  (3) $$\begin{array}{c} mtCP_{i-1}=\frac{\left(\;tCP_{i-1}+tCP_{i}\right)}{2}\text{ and }mtCP_{i}\;=\frac{\left(\;tCP_{i}+tCP_{i+1}\right)}{2}. \end{array}$$
(2) Especially, the first *Seg*_1_ and the last *Seg*_*n*_ can be presented according to the *tCP*_1_ and *tCP*_*n*_ as follows:
  (4) $$\begin{array}{c} Seg_{1}=\left\{X_{s},\ldots ,\;tCP_{1}\right\}\text{ and }Seg_{n}=\left\{tCP_{n},\ldots ,\;X_{e}\;\right\}, \end{array}$$
   where *X*_*s*_ and *X*_*e*_ are the two endpoints in *X*′, respectively.
(3) Then, the time series *X*′={*X*_*s*_,…, *X*_*j*_,…, *X*_*e*_} can be divided into a set of data segments  *SEG* set_*X*′_={*Seg*_1_,…,  *Seg*_*n*_ }. That is, *X*′={*Seg*_1_,…,  *Seg*_*n*_ }, and the following equation holds
  (5) $$\begin{array}{c} N_{X^{\prime }}=\overset{n}{\underset{i=1}{\sum }}N\_Seg_{i}, \end{array}$$

where *N*_*X*′_ is the total length of *X*′, and *N*_*Seg*_*i*_ refers to the size of *Seg*_*i*_.

The article "A Weighted Error Distance Metrics (WEDM) for Performance Evaluation on Multiple Change-Point (MCP) Detection in Synthetic Time Series" was published in 2022. Journal: Comput Intell Neurosci.

### 2.2. NED Evaluation on Single CP Detection

In the scheme of error distance (ED) measurement on single CP detection (Figure 2), each segment *Seg*_*i*_={*X*_*a*_ … *X*_*c*_ … *X*_*b*_} in time series *X*′={*Seg*_1_,…,  *Seg*_*n*_ } is divided into the former (left) part {*X*_*a*_,…, *X*_*c*−1_} and the latter (right) part {*X*_*c*+1_,…, *X*_*b*_} by the actual *tCP*_*i*_ located at the data point *X*_*c*_ and 1 ≤ *i* ≤ *n*.

From a statistical point of view, we refer to the former (left) part as a positive area and the latter (right) part as a negative one. When applying a CPD to detect the actual *tCP*_*i*_ in the data segment *Seg*_*i*_, a resultant *eCP*_*i*_ might be estimated from either the positive area or the negative one. A few concepts are introduced here to measure CPD model performance: true-positive distance (*tPD*), positive-error distance (*pED*), true-negative distance (*tND*), and negative-error distance (*nED*). If the resultant *eCP*_*i*_ is detected on the left side of the *tCP*_*i*_ (positive area), then *pED*_*i*_ and *tPD*_*i*_ can be calculated. That is, the distance from the *eCP*_*i*_ to the *tCP*_*i*_ and the start point, respectively. Meanwhile, *nED*_*i*_ and *tND*_*i*_ are not applicable. Conversely, when the *eCP*_*j*_ is estimated from the right side of the *tCP*_*i*_ (negative area), *nED*_*i*_ equals the distance from *eCP*_*j*_ to *tCP*_*i*_, and *tND*_*i*_ is the distance from the *eCP*_*j*_ to the end of the data segment *Seg*_*i*_. At the same time, *pED*_*i*_ and *tPD*_*i*_ do not exist (Figure 2). These definitions can be represented in formulas (6)–(9)as follows:

(6) $$\begin{array}{c} tPD_{i}=eCP_{i}\;-mCP_{i}\\ =X_{d}-X_{a}, \end{array}$$

(7) $$\begin{array}{c} pED_{i}=\;tCP_{i}\;-eCP_{i}\\ =X_{c}-X_{d},\\ =X_{b}-X_{e},\\ =X_{e}-X_{c}. \end{array}$$

(8) $$\begin{array}{c} tND_{i}=mCP_{i+1}-eCP_{j}\\ =X_{b}-X_{e},\\ =X_{e}-X_{c}. \end{array}$$

(9) $$\begin{array}{c} nED_{i}=eCP_{j}\;-tCP_{i}\;\\ =X_{e}-X_{c}. \end{array}$$

In which, *X*_*a*_ and *X*_*b*_ represent the start and endpoints of the time-series segment *Seg*_*i*_, respectively, *X*_*c*_ is the position of actual *tCP*_*i*_ in the  *Seg*_*i*_, *X*_*d*_ and *X*_*e*_ refer to the positions of resultant eCP on the left or right side of the *tCP*_*i*_ respectively.

The article "A Weighted Error Distance Metrics (WEDM) for Performance Evaluation on Multiple Change-Point (MCP) Detection in Synthetic Time Series" was published in 2022. Journal: Comput Intell Neurosci.

Basically, for a current data segment *Seg*_*i*_ in the scheme of NED evaluation on single CP detection (Figure 3), the distance between the start point and the *tCP*_*i*_ and the distance from the *tCP*_*i*_ to the end of each segment are both normalized to 1, and the normalized tCP position for each segment will match to the same point. In formulas (10)–(13),  *tPDR*_*i*_,  *pEDR*_*i*_,  *tNDR*_*i*_, and  *nEDR*_*i*_ can be interpreted as the normalized true-positive distance (*NtPD*_*i*_), normalized positive-error distance (*NpED*_*i*_), normalized true-negative distance (*NtND*_*i*_), and normalized negative-error distance (*NnED*_*i*_), respectively.

(10) $$\begin{array}{c} tPDR_{i}\left(NtPD_{i}\right)=\frac{\;tPD_{i}}{\;tPD_{i}\;+\;pED_{i}\;}, \end{array}$$

(11) $$\begin{array}{c} \;pEDR_{i}\left(NpED_{i}\right)=\frac{\;pED_{i}}{\;tPD_{i}\;+\;pED_{i}\;}, \end{array}$$

(12) $$\begin{array}{c} \;tNDR_{i}\left(NtND_{i}\right)=\frac{\;tND_{i}}{\;tND_{i}\;+nED_{i}\;}, \end{array}$$

(13) $$\begin{array}{c} nEDR_{i}\left(NnED_{i}\right)=\frac{\;nED_{i}}{\;tND_{i}\;+nED_{i}\;}. \end{array}$$

Thereafter, a normalized error distance *NED*^*i*^ in formula (14) is presented by a piecewise function of *NpED*_*i*_ and *NnED*_*i*_, according to the resultant *eCP*_*i*_ located at the positive or negative area.

(14) $$\begin{array}{c} NED^{i}=\left\{\begin{array}{cc} NpED_{i}, & e\;-CP_{i}\text{ on positive area},\;\\ NnED_{i}, & e\;-CP_{i}\text{ on negative area}. \end{array}\right) \end{array}$$

#### 2.2.1. WED Evaluation on MCPs Detection

Given a series of data segments *SEG* set_*X*′_ ={*Seg*_1_,…,  *Seg*_*n*_ } in a diagnosed time series *X*′ above, we can assemble all the resultant eCPs into an identical coordinate and present their NED  values ranging from the positive area [−1, 0] to the negative area [0, 1] in the *x*-axis (Figure 4). Then, the frequencies of *NED*^*i*^ can be defined in the all resultant eCPs as follows:

(15) $$\begin{array}{c} Freq\left(NED^{i}\;\right)=\frac{\text{Num}\left(NED^{i}\;\right)}{Nt}. \end{array}$$

In which, Num(*NED*^*i*^ ) is the number of the resultant eCPs that their NED values equal to *NED*^*i*^, and *Nt* is the number of resultant eCPs in total, 1 ≤ *i* ≤ *Nt*.

The article "A Weighted Error Distance Metrics (WEDM) for Performance Evaluation on Multiple Change-Point (MCP) Detection in Synthetic Time Series" was published in 2022. Journal: Comput Intell Neurosci.

Then, the weighted error distance *WED*^*i*^ is introduced according to the *NED*^*i*^ and *Freq*(*NED*^*i*^) in the resultant eCPs (Figure 5). For each *eCP*_*i*_ in the scattered distribution of resultant eCPs, its corresponding *WED*^*i*^ is equal to *WpED*_*i*_ or *WnED*_*i*_ depending on whether the *NED*^*i*^ is located at the positive-NpED or negative-NnED area ranging from −1 to 1 in the *x*-axis. The definitions of *WpED*_*i*_, *WnED*_*i*_, and *WED*^*i*^ are formulated as follows:

(16) $$\begin{array}{c} WpED_{i}\;=Freq\left(NpED_{i}\right)*NpED_{i},\\ WnED_{i}=Freq\left(NnED_{i}\right)*NnED_{i},\\ WED^{i}=\left\{\begin{array}{cc} WpED_{i}, & NED^{i},\;\text{on,}\;NpED\text{ area,}\\ WnED_{i} & NED^{i},\;\text{on,}\;NnED\text{ area}. \end{array}\right) \end{array}$$

Thereafter, a mean weighted error distance (*MWED*) is defined as follows:

(17) $$\begin{array}{c} MWED=\frac{\sum_{i=1}^{l}WPED_{i}+\sum_{j=1}^{r}WNED_{j}}{l\;+r}, \end{array}$$

where *l* and *r* refer to the numbers of the *eCPs* located before and after the actual tCP*s* (positive-NpED area and negative-NnED area), respectively. In most of the CPD models, when the search algorithm reaches the start or end of the time series, if no change point is found, then the resultant eCP can be set as either the start or the end. Therefore, the sum of *l* and *r* will be equal to *N* (the total number of actual tCPs to be diagnosed in a time series *X*′). Formula (17) can be simplified as follows:

(18) $$\begin{array}{c} MWED=\frac{\sum_{i=1}^{N}WED_{i}}{N}. \end{array}$$

Furthermore, following MWED, 1-MWED can be referred to as mean weighted true distance (MWTD) and used as a measure of the overall performance of a CPD model for MCPs detection on time series with a series of data fluctuations.

## 3. Results and Discussion

To accurately evaluate different CPD models, other related indexes were introduced besides our WEDM. In the synthetic experiments, time-series datasets were generated and assembled by using the Gaussian distribution function in the Matlab platform, and then repetitive tests on single CP detection were executed by using different TST, BST, KS, and SSA models. Meanwhile, the performance of CPD models was evaluated by using successive tests on MCPs detection that were implemented under different RSW and FSW frameworks, respectively.

The article "A Weighted Error Distance Metrics (WEDM) for Performance Evaluation on Multiple Change-Point (MCP) Detection in Synthetic Time Series" was published in 2022. Journal: Comput Intell Neurosci.

### 3.1. Related Evaluation Indexes

In the synthetic tests, some other indexes are used for evaluating the convergence of different CPD models, including the hit, miss, and error rates, and computing time. Given a data segment *Seg*_*i*_ in the time series *X*' mentioned above, the related definitions are introduced in terms of the error distance between the resultant *eCP*s and the actual *tCP*_*i*_ as follows (Figure 6):

(1) *Error distance*: Given an actual tCP_*i*_ assigned in the current data segment *Seg*_*i*_, the error distance *ED*_*tCPi*_ between each pair of the estimated *eCP*_*j*_ and the *tCP*_*i*_ is defined by *ED*_*tCPi*_=|*eCP*_*j*_ − *tCP*_*i*_|.
(2) *Hit area*: For the actual *tCP*_*i*_, the hit area named *HA*_*tCPi*_ is formulated by *HA*_*tCPi*_=[*tCP*_*i*_  − *hd*_*i*_, *tCP*_*i*_ +*hd*_*i*_], where *hd*_*i*_ is the threshold value of error distance between *tCP*_*i*_ and *eCP*_*j*_.
(3) *Hit*: Given an error distance *ED*_*tCPi*_ mentioned above, if 0 ≤ *ED*_*tCPi*_ ≤ *hd*_*i*_ holds, then the *tCP*_*i*_ is hit by *eCP*_*j*_ and recorded by Hit(*tCP*_*i*_)=1. Therefore, the value of *WED*^*i*^ defined in formula (18) equals 0.
(4) *Error*: On the other hand, if *ED*_*tCPi*_ > *hd*_*i*_ holds, then *eCP*_*j*_ is dealt as an error result labeled by Error(*eCP*_*j*_)=1. In this circumstance, the value of *WED*^*i*^ is within the rage (0,  1).
(5) *Miss*: In addition, if no change point is detected from the *Seg*_*i*_, then the target *tCP*_*i*_ is missed, and identified by Miss(*tCP*_*i*_)=1. Accordingly, the value of *WED*^*i*^ is set to be 1 because of the missing *tCP*_*i*_.
Thereafter, the hit rate, miss rate, and error rate are formulated as follows:
  (19) $$\begin{array}{c} \text{Hit rate}=\left(\frac{N_{hit}}{N_{eCPs}}\right)*100\%,\\ \text{Miss rate }=\;\left(\frac{N_{miss}}{N_{eCPs}}\right)*100\%,\\ \text{Error rate}=\left(\frac{N_{error}}{N_{eCPs}}\right)*100\%. \end{array}$$
In which, *N*_hit_=∑_*i*=1_^*N*_*tCPs*_^Hit(*tCP*_*i*  _) is the number of actual tCPs hit by the resultant eCPs, *N*_Miss_=∑_*i*=1_^*N*_*tCPs*_^Miss(*tCP*_*i*  _) is the part of actual tCPs that are missed, and *N*_Error_=∑_*i*=1_^*N*_*tCPs*_^Error(*eCP*_*i*  _) stand for the number of the resultant *MCPs* in which *D*_*tCPi*_ > *hd*_*i*_ holds. *N*_*eCPs*_ is the number of resultant *MCPs* in total, and it is usually larger than *N*_*tCPs*_, that is, the number of the actual tCPs within the time series *X*′ . Generally, it holds true that hit rate + miss rate + error rate =1 for all the resultant eCPs.
(6) *Computing time*: In addition, for a certain CPD model *k*, the computing time is mainly used for tCPs detecting from the multiple data segments in *X*′, and it can be denoted as follows:
  (20) $$\begin{array}{c} ST^{k}=\overset{N_{s}}{\underset{i=1}{\sum }}ST_{i}, \end{array}$$

where *ST*_*i*_ refers to the computing time cost in the *Seg*_*i*_, and *N*_*s*_  is the total data segments. Then, the normalized time is defined as follows:

(21) $$\begin{array}{c} NST^{k}=\frac{ST^{k}}{\sum_{k=1}^{n}ST^{k}}. \end{array}$$

In which, *ST*^*k*^ stands for the computing time of the model *k*, and *n* is the total model to be compared. The  *NST*^*k*^ represents the time ratio of model *k* to all methods, and then it can reflect the searching efficiency against others. Generally, both TST and BST models in our previous studies have a time complexity of nearly *O*(log *N*) [8, 10, 13]; therefore, they should be faster and more efficient than some traditional algorithms with time complexity about *O*(*N*^2^), such as KS, CUSUM, *t*-test, or SSA methods.

The article "A Weighted Error Distance Metrics (WEDM) for Performance Evaluation on Multiple Change-Point (MCP) Detection in Synthetic Time Series" was published in 2022. Journal: Comput Intell Neurosci.

### 3.2. Repetitive Tests on Single CP Detection

In the first experiment, repetitive tests on single CP detection were executed on the synthetic dataset, that is, Dataset1 ={*X*^1^,…*X*^*i*^,…, *X*^*K*^} that was generated by the Gaussian function in the Matlab R2016 platform. For each time series *X*^*i*^={*x*_1_,   …, *x*_*i*_,   …  *x*_*N*_} with single target CP, it is composed of both the positive area *X*^*iL*^={*x*_1_,   …,  *x*_*m*_} and the negative area *X*^*iR*^={*x*_*m*+1_,   …,  *x*_*N*_} before and after the assigned target *tCP*_*i* _=*x*_*m*_. The former *X*^*iL*^ and latter *X*^*iR*^ were generated by the normal distribution *N* (*μ* = 0, *σ* = 1) of size *m* (*m* time points included in the positive area), and *N* (*μ* = *V*, *σ* = 1) of size *N*-*m* (*N-m* time points in the negative area), respectively, where *V* is a constant mean value, and *N* is the total length of *X*^*i*^.

Here, we first present the results from Dataset1 that was composed of multiple 20 data groups with different length *N*, variance *V*, and *tCP*, and each group contains 100 time-series samples. Therefore, Dataset1 included 2000 time series in total, and this experiment named Exp1 is performed by using TST, BST, KS, T, and SSA models, respectively. In our simulations, the time-series samples in each group were generated by selecting the random values of sample length *N* from 2^10 to 2^15, variance *V* from 1.0 to 3.7, and the position of actual *tCP* from 1 to *N*.

In the 20 groups of Exp1, the repetitive tests are executed by using different CPD models including the TST, BST, KS, T, and SSA, respectively (Figure 7). With the total 2000 time-series samples in Dataset1, the frequency and WED distribution of resultant MCPs are illustrated from the positive-NpED range of [−1, 0] to the negative-NnED range of [0, 1] in the *x*-axis. From these results, we can see that if the resultant eCP is much closer to the central axis of *x* = 0, then the WED value generally gets smaller and tends to be 0, and vice versa. In all five models, TST and KS obtain the eCPs that are mostly located near the central field of *x* = 0, and then have narrower WED distributions and smaller WED values than other models, except that TST has a few eCPs fallen into the positive-NpED field. As for other BST, T, and SSA models, the eCPs are mainly scattered with a wide range from the NpED to the NnED areas, therefore their WED distributions are wider and bigger, especially for T and SSA.

The article "A Weighted Error Distance Metrics (WEDM) for Performance Evaluation on Multiple Change-Point (MCP) Detection in Synthetic Time Series" was published in 2022. Journal: Comput Intell Neurosci.

Meanwhile, these simulation results also illustrate that both TST and KS have better convergency than others, especially, the TST has the highest hit level and takes the shortest convergent time in all five models. For the rest models, BST seems much better than others, and T has the worst convergency, because of the lowest hit, the biggest error, and convergent time in all five models. Furthermore, the mean analyses (Table 1) indicate that the TST takes the shortest computing time, has the highest hit rate, the smallest MWED, and the biggest MWTD out of the other four models. For T and SSA models, a lot of eCPs are scattered the whole field from NPED to NNED, especially, T has the biggest values of error rate and MWED and needs the longest time in all five models.

In addition, the efficiencies of five models are evaluated using random parameter values in a total of 20 tests. The dynamic tracks including hit rate, miss rate, error rate, and MWED are illustrated versus the test number from 1 to 20 (Figure 8). Also, the mean analyses on hit rate, miss rate, error rate, and MWED are presented in the histograms, in which, “1,” “2,” “3,” “4,” and “5” in *x*-axis refer to the TST, BST, KS, T, and SSA models, respectively. In the whole process of simulation tests, the TST model has a relatively higher hit rate with some fluctuations and keeps more stable and lower levels of miss rate, error rate, and MWED than others. Although KS has a smaller hit rate than TST and BST, it keeps lower tracks of miss and error rates than BST, T, and SSA. To some extent, BST has a bigger hit rate, and lower values of error rate and MWED than T and SSA, it seems unstable due to the drastic oscillations in the tracks of hit and miss rates. For T and SSA, both models have smaller hit rates and keep dramatic fluctuations in the tracks of error rate and MWED value, despite a lower miss rate than BST.

The article "A Weighted Error Distance Metrics (WEDM) for Performance Evaluation on Multiple Change-Point (MCP) Detection in Synthetic Time Series" was published in 2022. Journal: Comput Intell Neurosci.

Furthermore, taking one representative test as an example, the simulations of single CP detection are repetitively executed by using 100 time-series samples with random values of parameters *N* *=* 2^14, *tCP* = 12267, and *V* = 1.9. For different TST, BST, KS, T, and SSA models, the resultant eCPs are illustrated using the locations, distributions, frequency, and WED, in line with the test number, time-series positions, NPED, and NNED in the *x*-axis, respectively (Figure 9). For both TST and KS models, it is easy to see that most of the eCPs are located within the small range near the actual *tCP* = 12267, and similar results can be found in the distribution, frequency, and WED analyses on the resultant eCPs. On the contrary, similar results for the rest of BST, T, and SSA models are that lots of the eCPs are randomly scattered across the fields from NPED to NNED, and small parts of the eCPs are gathered near the actual *tCP*.

Then, the mean analyses for this representative test are summarized in terms of WMTD, hit rate, miss rate, error rate, MWED, and time (Table 2). The results show that the TST model has much smaller values of MWED, miss and error rates, and computing time, as well as the biggest values of hit rate and MWTD than others. Despite a long time and smaller hit rate than TST, KS kept similar levels of MWTD, hit, miss, and error rates with it. As for the rest BST, T, and SSA, although the three models had similar performance, BST had the biggest miss rate, T had the smallest MWTD and hit rate, and the biggest values of time, error rate, and MWED.

#### 3.2.1. Successive MCPs Detection under the RSW Framework

In the second experiment, successive tests on MCPs detection were implemented by using other synthetic datasets such as Dataset2 ={*X*^1^,…*X*^*i*^,…, *X*^*W*^ } that was composed of *W* time-series samples, and each sample *X*^*i*^={*Seg*^1^,…,  *Seg*^*j*^,…*Seg*^*n*^ } was assembled by *n* data segments with different features and distributions. For a given *tMCP* set={*tCP*_1_,…, *tCP*_*n*_}, each *tCP*_*i*_ is assigned between two adjacent segments *Seg*^*i*^ and *Seg*^*i*+1^, 1 ≤ *i*≤*n* − 1. Then, the sample *X*^*i*^ can be denoted as *X*^*i*^  = {*x*_1_^*s*1^,…*x*_*Ns*1−1_^*s*1^, *tCP*_1_,…,  *x*_1_^*sj*^,…*x*_*Nsj*−1_^*sj*^, *tCP*_*j*_,  *x*_1_^*sn*^,…*x*_*Nsn*−1_^*sn*^, *tCP*_*n*_}, where *Nsj* is the size of segment *Seg*^*j*^ in *X*^*i*^. In the successive tests on MCPs detection, two experiments named Exp2 and Exp3 were implemented based on Dataset2 under the RSW and FSW frameworks, respectively. For each experiment, a series of tests for MCPs detection was executed by using TST, BST, KS, T, and SSA models, respectively.

The article "A Weighted Error Distance Metrics (WEDM) for Performance Evaluation on Multiple Change-Point (MCP) Detection in Synthetic Time Series" was published in 2022. Journal: Comput Intell Neurosci.

In Exp2, the number of segments *n* within each sample *X*_*i*_ was stochastically chosen from 15 to 30, and each data segment *Seg*_*j*_ = {*x*_1_^*sj*^,…,  *X*_*Nsj*_^*sj*^} was randomly generated by the Gaussian distribution *N*(*U*_*j*_, *V*_*j*_) of length *Nsj* from 2^12 to 2^15, with mean *U*_*j*_ from 1.0 to 0.1 × *N*_*MCPs*_, and variance *V*_*j*_ from 1 to 2.0 × *N*_*MCPs*_, respectively. Here, we present the results of successive tests on MCPs detection under the RSW framework. First, the frequency and WED distribution of resultant MCPs (Figure 10) are displayed within the whole range from the negative-NPED field to the positive-NNED field in the *x*-axis. Generally, for a certain CPD model, the resultant MCPs are closer to the central axis *x* = 0, their values of MWED are much smaller. In contrast, the bigger MWTD has, the better efficiency is, and vice versa. In all five models, the results (Figure 10) and the mean analyses (Table 3) show that most of the resultant MCPs detected by TST are located near the central axis *x* = 0, and TST has the biggest hit rate, the smallest values of miss and error rates, therefore it has the highest MWTD out of others. For the BST model, although a lot of the resultant MCPs are scattered away from the central axis *x* = 0, it has a smaller error rate and MWED, as well as a bigger hit rate and MWTD than the rest models. For KS, T, and SSA, the common feature is that most of the resultant MCPs are spread through the whole field ranging from −1 to 1 in the *x*-axis. KS has a bigger MWTD than the other two, T has the smallest MWTD, and SSA has the biggest values of error rate and computing time in all five models.

Meanwhile, these simulations illustrate that the TST has the best convergency because it has the highest hit level, the lowest error, and takes the shortest convergent time in all five models. For the others, the BST model has much better convergency due to the higher hit, lower error, and shorter time than others. SSA seems the worst one in all five models, because of the lowest hit, the biggest error, and convergent time.

Second, the performance of five CPD models is demonstrated by a series of 10 tests in total, in which the respective parameters of the sample size *N*, the number of MCPs *N*_*MCPs*_, the mean *μ*, and variance  *δ* are randomly taken from 2^12–2^15, 15∼30, 1∼0.1 × *N*_*MCPs*_, and 1∼2 × *N*_*MCPs*_, respectively. The results of dynamic tracks and mean analyses (Figure 11) indicate that the TST model still keeps a better grade with a higher and more stable level of hit rate, as well as the lower levels of error rate and MWED than the other four models. Although BST looks more efficient than KS, T, and SSA, the dynamic tracks in all four items present stronger fluctuations, especially for the miss rate. This probably means that BST has unstable performance during the process of MCPs detection. As for the rest models, they all have similar tracks of lower hit rate and bigger error rates. KS presents instability due to the fluctuant tracks of miss rate and MWED, and so does the T model because of the fluctuant miss rate in the total of random 10 tests. Also, the model's performance can be intuitively evaluated and distinguished from each other in terms of the mean analyses in the histograms (Figure 11(e)–11(h)).

The article "A Weighted Error Distance Metrics (WEDM) for Performance Evaluation on Multiple Change-Point (MCP) Detection in Synthetic Time Series" was published in 2022. Journal: Comput Intell Neurosci.

Last, one representative test is selected from Exp2 above, and the simulations of MCPs detection are demonstrated by using a time series with *nMCPs* *=* 25 (Figure 12). For the diagnosed data sample (Figure 12(f)), the distributions of resultant MCPs are illustrated by using different CPD models of TST, BST, KS, T, and SSA models, respectively (Figure 12(a)–12(e)). The results of frequency and WED distribution of resultant MCPs (Figure 13) and mean analyses (Table 4) reveal that the TST is a superior one in all five models because most of the resultant MCPs hit the target MCP positions, and few of them are dealt with as miss or error states. The BST model takes second place due to a smaller hit rate and bigger error rate than TST. For the rest models, KS, T, and SSA get worse one by one because more numbers of resultant MCPs are in the error state. As a result, the hit rate gets lower, and MWED takes bigger as well.

Successive MCPs detection under the FSW framework.

In the Exp3 under the FSW framework, the total of 30 data segments was arranged within each sample *X*_*i*_, and each data segment *Seg*_*j*_ = { *x*_1_^*sj*^,…,  *X*_*Nsj*_^*sj*^} was randomly generated by the Gaussian distribution *N*(*U*_*j*_, *V*_*j*_) of length *N*_*sj*_ from 2^12 to 2^15, with mean *U*_*j*_ from 1.0 to 0.1 × 30 and variance *V*_*j*_ from 1 to 2.0 × 30, as well as with the size of fixed slide window *N*_*fsw*_ ranging from 2^6 to 2^15, respectively.

In our simulations, we execute a total of 10 successive tests on MCPs detection under the FSW framework. First, the frequency and WED distribution of resultant MCPs (Figure 14) are displayed from the negative-NPED field to the positive-NNED field in the *x*-axis. Generally, for a certain CPD model, the resultant MCPs are much closer to the central axis *x* = 0, and their WED values are much smaller. The results (Figure 14 and Table 5) indicate that for the TST model, most of the resultant MCPs detected are located near the central axis *x* = 0, and it has the biggest hit rate, the smallest values of error rate, MWED, and computing time; therefore, it has the highest MWTD in all five CPD models. As for BST, KS, T, and SSA models, the common feature is that most of the resultant MCPs are randomly scattered through the whole field ranging from −1 to 1 in the *x*-axis. For KS, it has a smaller miss rate and MWED and a bigger MWTD than the others. Although BST has a bigger hit rate and shorter time, it has a bigger MWED and smaller MWTD than TST and KS. T and SSA have much bigger values of MWED, error rate, and smaller MWTD, especially SSA has the smallest MWTD and the biggest values of error rate and time in all five models.

The article "A Weighted Error Distance Metrics (WEDM) for Performance Evaluation on Multiple Change-Point (MCP) Detection in Synthetic Time Series" was published in 2022. Journal: Comput Intell Neurosci.

Meanwhile, these simulations illustrate that the TST has the best convergency, in terms of the highest hit, the lowest error, and the shortest time in all five models. For the other four models, the BST model is much better than the rest ones, because it has a relatively higher hit level, lower error rate, and much shorter time than others. Unfortunately, SSA has the worst convergency in all five models, due to the lowest hit level, the biggest error rate, and the longest convergent time out of the other four models.

Second, the performance evaluation on five CPD models is demonstrated respectively by a series of successive MCPs detection tests in Exp3. Generally, the dynamic tracks and histogram analyses (Figure 15) show that all five CPD models present respective instability in response to the size of the fixed slide window, *N*_*fsw*_ ranging from 2^6 to 2^15, especially for the TST, BST, and KS models. Despite the TST model having the biggest miss rate with drastic fluctuations, it still keeps a better efficiency due to the highest hit rate and the lowest levels of error rate and MWED out of the other four models. As for the rest ones, BST seems better than KS, T, and SSA, because of the higher hit rate and the slightly decreasing level of error rate. Although KS reversely keeps decreasing hit rate and increasing error rate with big fluctuation, it seems better than T and SSA, on account of lower levels of miss rate and MWED. Both T and SSA present inefficiency and insensitivity in response to the increasing *N*_*fsw*_, especially for the SSA model, with the lowest hit rate and the highest levels of error rate and MWED out of other ones.

Last, taking the TST model as an example, five representative simulations are selected from the total 10 tests in the FSW framework of Exp3 (Figure 16(a)–16(e)), and then the performance evaluation is listed under the values of *N*_*fsw*_ = 2^6, 2^8, 2^12, 2^14, and 2^15, respectively (Table 6). Given one data sample with *N*_*MCPs*_ = 30 (Figure 16(f)), the results of MCPs detection show that the TST model presents the best performance as *N*_*fsw*_ = 2^12, in terms of the biggest values of hit rate and MWTD, and the smallest values of miss and error rates and MWED in all five tests. However, the efficiency of TST tends to be worse as the value of *N*_*fsw*_ takes too bigger or too smaller. Therefore, the size of the fixed slide window is a key factor for the FSW framework during the MCPs detection.

The article "A Weighted Error Distance Metrics (WEDM) for Performance Evaluation on Multiple Change-Point (MCP) Detection in Synthetic Time Series" was published in 2022. Journal: Comput Intell Neurosci.

In all, these results in the two experiments above suggest that the proposed WED method can visually present the distribution of resultant eCPs in the error state and the normalized distance from the target position of zero in the *x*-axis. The simulation results suggest that the mean analyses of MWED can generally count the mean value of error ratio against total tests and then measure the efficiency of a certain model in the successive MCPs detection. The performances of different CPD models can be evaluated, and the better ones can be discerned from the others.

## 4. Conclusions and Discussion

In this study, a novel WEDM method is proposed for evaluating the overall performance of a CPD model across not only repetitive tests on single CP detection, but also successive tests on multiple change-point (MCP) detection on synthetic time series under different RSW and FSW frameworks. In this WEDM method, a concept of normalized error distance was introduced that allows comparisons of the distance between the estimated change-point (eCP) position and the target change-point (tCP) in the synthetic time series. Especially, both positive- and negative-error distances between resultant eCPs and actual tCPs are weighted or normalized for creating WED metrics.

As opposed to previous methods, our WEDM allows comparison when CPD is used across multiple time-series samples with different lengths and variances, especially cross multiple data segments in an identical time series, with different patterns, such as data distributions, segment sizes, and number and positions of targets tCPs. In the successive MCPs detection, our WEDM method first divides the original sample into a series of data segments in terms of assigned target change points and then calculates a normalized error distance (NED) value for each segment. Next, WEDM presents the frequency and WED distribution of the resultant eCPs from all data segments in the normalized positive-error distance (NPED) and the normalized negative-error distance (NNED) intervals in the same coordinates. Last, the mean WED (MWED) and MWTD (1-MWED) were obtained and dealt with as important performance indexes.

The article "A Weighted Error Distance Metrics (WEDM) for Performance Evaluation on Multiple Change-Point (MCP) Detection in Synthetic Time Series" was published in 2022. Journal: Comput Intell Neurosci.

In our simulations, a series of MCPs detection tests were executed by using synthetic time-series datasets in the Matlab platform, and the proposed method was applied to the evaluation of the CPD utilizing TST, BST, KS, T, and SSA models under repetitive single CP detection in Exp1, successive MCPs detection under the RSW in Exp2, and FSW framework in Exp3, respectively. The results of the study showed its ability to compare the results from the CPD models working with a series of synthetic tests on multiple time-series samples. The WED metrics offer a new way of evaluating CPD performance. It allows better visualization of the distribution of the resultant eCPs when the CPD models work on multiple time series with different data features, as well as multiple data segments of a time-series sample with different data patterns. Meanwhile, the convergence of different CPD models was analyzed in terms of the dynamic tracks and mean analyses on the value of WED, as well as other measurements, including the rates of hit, error, and miss, and the computational cost. Our WEDM method can not only offer a visualizable and overall measure but also give better advice for users as to what CPD models to use based on the application.

## Figures and Tables

**Figure 1:** The scheme of WEDM evaluation on the target MCPs detection in the diagnosed *X*′.

**Figure 2:** The scheme of error distance (ED) measurement on single CP detection in the data segment *Seg*_*i*_. In the positive area, *X*_*a*_ represents the start point of *Seg*_*i*_, and *X*_*d*_ is the position of resultant *eCP*_*i*_ within the positive area before the actual *tCP*_*i*_. On the other hand, *X*_*b*_ represents the endpoint of *Seg*_*i*_, and *X*_*e*_ stands for the *eCP*_*j*_ located within the negative area after the *tCP*_*i*_.

**Figure 3:** The scheme of NED evaluation on single CP detection in the data segment *Seg*_*i*_. In which, “−1” and “1” represent the start and endpoints of *Seg*_*i*_, and “0” refers to the position of actual *tCP*_*i*_ in the *x*-axis, respectively.

**Figure 4:** The scheme of *NED* evaluation for MCPs detection on *tMCPset* =  {*tCP*_1_,…, *tCP*_*m*_} in a time series *X*′. For each resultant *eCP*_*i*_, the value of *NED*^*i*^ equals to *NpED*_*i*_ or *NnED*_*i*_ depending on that the *eCP*_*i*_ is located at the positive or negative area ranging from −1 to 1 in the *x*-axis.

**Figure 5:** The scheme of WED metrics for MCPs detection on a set of target MCPs *tCPset* =  {{*tCP*_1_,…, *tCP*_*m*_} in a time series *X*′. For each *eCP*_*i*_ in the scattered distribution of resultant eCPs, the value of *WED*^*i*^ refers to *WPED*_*i*_ or *WNED*_*i*_ according to whether the *NED*^*i*^ is located at the positive-NpED or negative-NnED area ranging from −1 to 1 in the *x*-axis.

The article "A Weighted Error Distance Metrics (WEDM) for Performance Evaluation on Multiple Change-Point (MCP) Detection in Synthetic Time Series" was published in 2022. Journal: Comput Intell Neurosci.

**Figure 6:** The scheme of single CP detection on the data segment *Seg*_*i*_  within a sliding window Wi. The definitions of hit, error, miss, and redundant are introduced according to the distance between tCP and eCP, respectively.

**Figure 7:** The frequency and WED distribution of resultant MCPs from the 20 groups in Dataset1. For the different models of (a) TST, (b) BST, (c) KS, (d) T, and (e) SSA, the frequency and WED distribution of the resultant MCPs are demonstrated from the NpED range of [−1, 0] to the NnED range of [0, 1] in the *x*-axis, respectively.

**Figure 8:** The results of multiple 20 tests on single CP detection by using 2000 synthetic time series in Dataset1 of Exp1, with random parameters of sample size (N) from 2^10 to 2^15, actual *tCP* from start to end of sample length (N), and variance (V) from 1.0 to 3.7. For TST, BST, KS, T, and SSA models, the dynamic tracks of (a) hit rate, (b) miss rate, (c) error rate, and (d) MWED versus simulation tests range from 1 to 20. In addition, the mean analyses on (e) hit rate, (f) miss rate, (g) error rate, and (h) MWED, in which, “1” “2”, “3”, “4”, and “5” in *x*-axis refer to the TST, BST, KS, T, and SSA models, respectively.

**Figure 9:** The repetitive simulations of single CP detection on 100 time series from one of 10 tests in Exp1, with random parameter values of sample size *N* *=* 2^14, actual *tCP* = 12267, and variance (V) = 1.9. By using different TST, BST, KS, T, and SSA models, the simulation results including (a) locations, (b) distributions, (c) frequency, and (d) WED of the resultant eCPs are represented in line with the test number, time-series positions, NPED, and NNED in the *x*-axis, respectively.

**Figure 10:** The analyses on the frequency and WED distribution of resultant MCPs in the total 10 tests of Exp2. For the different MCP models of (a) TST, (b) BST, (c) KS, (d) T, and (e) SSA under the RSW framework, the frequency and WED distribution of resultant MCPs are illustrated within the NPED ranging from −1 to 0, and the NNED ranging from 0 to 1 in the *x*-axis.

**Figure 11:** The simulations of MCPs detection on the total of 10 tests in Exp2 under the RSW framework, with random parameters of sample size *Nsj* from 2^12 to 2^15, the number of tCPs *N*_*MCPs*_ from 15 to 30, mean *U*_*j*_ from 1 to 0.1 × *N*_*MCPs*_, and variance *V*_*j*_ from 1 to 2 × *N*_*MCPs*_, respectively. For the different TST, BST, KS, T, and SSA models, the performance analyses are denoted in (a) hit rate, (b) miss rate, (c) error rate, and (d) MWED, respectively. Furthermore, the mean analyses are illustrated in histograms of (e) hit rate, (f) miss rate, (g) error rate, and (h) MWED, in which, “1,” “2,” “3,” “4,” and “5” in *x*-axis refer to TST, BST, KS, T, and SSA, respectively.

The article "A Weighted Error Distance Metrics (WEDM) for Performance Evaluation on Multiple Change-Point (MCP) Detection in Synthetic Time Series" was published in 2022. Journal: Comput Intell Neurosci.

**Figure 12:** The simulations of MCPs detection on the representative test with *N*_*MCPs*_ = 25. For one selected sample in (f), the resultant MCPs are illustrated by using different models of (a) TST, (b) BST, (c) KS, (d) T, and (e) SSA, respectively.

**Figure 13:** The results of WED evaluation on the 100 samples with *N*_*MCPs*_ = 25 in Exp2. For the different MCP models of (a) TST, (b) BST, (c) KS, (d) T, and (e) SSA, the frequency and WED distribution of resultant MCPs are illustrated within the NPED ranging from −1 to 0, and the NNED ranging from 0 to 1 in the *x*-axis, respectively.

**Figure 14:** The analyses on the frequency and WED distribution of resultant MCPs in the total 10 tests of Exp3. For the different MCP models of (a) TST, (b) BST, (c) KS, (d) T, and (e) SSA under the FSW framework, the frequency and WED distribution of resultant MCPs are illustrated within the NPED field ranging from −1 to 0 and the NNED field ranging from 0 to 1 in the *x*-axis.

**Figure 15:** The simulations of MCPs detection on the total of 10 tests in Exp3 under the FSW framework, with random parameters of sample size *N*_*sj*_ from 2^12 to 2^15, the fixed number of tCPs *N*_*MCPs*_ = 30, mean *U*_*j*_ from 1 to 0.1 × 30, and variance *V*_*j*_ from 1 to 2 × 30, respectively. For the different CPD models of TST, BST, KS, T, and SSA, the performance analyses are denoted in (a) hit rate, (b) miss rate, (c) error rate, and (d) mwed, respectively. Furthermore, the mean analyses are illustrated in (e) hit rate, (f) miss rate, (g) error rate, and (h) MWED, in which, “1,” “2,” “3,” “4,” and “5” in *x*-axis refer to TST, BST, KS, T, and SSA, respectively.

**Figure 16:** The simulations of MCPs detection by TST model under different sizes of fixed slide window *N*_*fsw*_ in the FSW framework. Given the diagnosed data sample with *N*_*MCPs*_ = 30 in (f), the resultant MCPs detection is illustrated under different *Nfsw* values of (a) 2^6, (b) 2^8, (c) 2^12, (d) 2^14, and (e) 2^15, respectively.

**Table 1:** The mean analyses of single CP detection in Exp1 by using TST, BST, KS, T, and SSA models.

Items	Methods				
	TST	BST	KS	T	SSA
MWTD	0.9972	0.9633	0.9947	0.7030	0.8349
Hit rate	0.4040	0.1540	0.0430	0.0340	0.0585
Miss rate	0.0005	0.0035	0.0000	0.0005	0.0005
Error rate	0.0012	0.0038	0.0002	0.1202	0.0601
MWED	0.0028	0.0367	0.0053	0.2970	0.1651
Time	0.0032	0.0039	0.3126	0.5239	0.1566

The article "A Weighted Error Distance Metrics (WEDM) for Performance Evaluation on Multiple Change-Point (MCP) Detection in Synthetic Time Series" was published in 2022. Journal: Comput Intell Neurosci.

**Table 2:** The analyses of one representative test on repetitive single CP detection by different CPD models.

items	Methods				
	TST	BST	KS	T	SSA
MWTD	**0.9998**	**.7315**	**0.9980**	**0.5708**	**0.6567**
Hit rate	0.3400	0.0600	0.0400	0.0010	0.0020
Miss rate	0.0000	0.0001	0.0000	0.0000	0.0000
Error rate	0.0001	0.0259	0.0001	0.2496	0.1536
MWED	0.0002	0.2685	0.0020	0.4292	0.3433
Time	0.0012	0.0012	0.3276	0.5861	0.0840

**Table 3:** The performance analyses on MCPs detection by five CPD models in Exp2 under the RSW framework.

items	Methods				
	TST	BST	KS	T	SSA
MWTD	**0.9264**	**0.8856**	**0.7850**	**0.5141**	**0.5299**
Hit rate	0.8629	0.6255	0.2256	0.2029	0.0820
Miss rate	0.0398	0.0585	0.0430	0.0471	0.0018
Error rate	0.1006	0.3421	0.7682	0.7661	0.8851
MWED	0.0736	0.1144	0.2150	0.4859	0.4701
Time	0.0004	0.0003	0.1483	0.1134	0.7376

**Table 4:** The mean analyses on five CPD models in one representative MCPs detection test with *N*_*MCPs*_ = 25.

items	Methods				
	TST	BST	KS	T	SSA
MWTD	**0.9655**	**0.9319**	**0.8836**	**0.6042**	**0.5779**
Hit rate	0.9310	0.5667	0.3030	0.2222	0.0727
Miss rate	0.0345	0.0333	0.0303	0.0635	0.0000
Error rate	0.0345	0.4333	0.6970	0.7619	0.8909
MWED	0.0345	0.0681	0.1164	0.3958	0.4221
Time	0.0004	0.0003	0.1889	0.1209	0.6896

**Table 5:** The mean analyses on MCPs detection in Exp3 by five CPD models under the FSW framework.

Items	Methods				
	TST	BST	KS	T	SSA
MWTD	**0.9875**	**0.7758**	**0.8268**	**0.5063**	**0.5009**
Hit rate	0.7867	0.5167	0.3106	0.1862	0.0525
Miss rate	0.1900	0.0930	0.0894	0.0977	0.0633
Error rate	0.0200	0.4186	0.6194	0.7271	0.9004
MWED	0.0125	0.2242	0.1732	0.4937	0.4991
Time	0.0006	0.0008	0.1419	0.0766	0.7802

**Table 6:** The performance evaluations on the TST model with different *N*_*fsw*_ under the FSW framework in Exp3.

Items *N*_*fsw*_ *=*	Hit rate	Miss rate	Error rate	MWED	MWTD
2^6	0.4667	0.5333	0.0000	0.5333	0.4667
2^8	0.7000	0.3000	0.0000	0.3000	0.7000
**2^12**	**0.9667**	**0.0303**	**0.0333**	**0.0586**	**0.9414**
2^14	0.7667	0.2000	0.0333	0.2002	0.7998
2^15	0.6000	0.3333	0.0000	0.3333	0.6667

## Data Availability

Some synthetic time-series datasets were generated in the Matlab simulation platform, and no real datasets are used specially for the experimental validations in this study.
